# An Exploration of the Differences between Chinese and Western Costumes in the Archaeological Archaeology of Clothing Culture in Different Periods of Agriculture

**DOI:** 10.1155/2022/2491990

**Published:** 2022-06-15

**Authors:** Jiwen Zhang

**Affiliations:** School of New Media Art, Xi'an Polytechnic University, Xi'an 710048, China

## Abstract

Countries around the world have different historical development processes in different periods of agricultural economic environment, and have formed different costume culture characteristics. This study analyzes the differences in aesthetic standards in Chinese and Western clothing cultures, as well as the differences between Chinese and Western costumes in color design, structural design, and dress methods, and elaborates the main reasons for the differences between Chinese and Western clothing cultures. The study focuses on the characteristics and differences of traditional clothing art culture in various places, but because of the differences in historical conditions, lifestyles, psychological qualities, and traditional ideas and cultural concepts, there are great differences between the traditional costume art culture concepts in China and the West. Based on this, the study specifically explains the difference between the two through the comparison of the aesthetic characteristics of the traditional costume art culture concepts in the Middle East and the West, and the difference in the expression of the Middle East and Western clothing art.

## 1. Introduction

China's costume culture can be traced back to 5,000 years ago, and each dynasty and historical period is full of distinctive characteristics. Traditional Chinese costumes are mainly Hanfu, Hufu, and flag costumes [1]. Western costume culture can be traced back to Mesopotamia and Egypt. The history is also very long. Because of different cultures, different histories, and different environments, the external manifestations of Western and Chinese clothing are also different, and they are all an indispensable part of the history of human clothing [2]. Clothing is like a mirror, which illuminates the different historical and cultural backgrounds and connotations of various countries and regions. The difference between Chinese and Western clothing has a certain relationship with the cultural differences between China and the West, and the cultural differences between Chinese and Western clothing are actually the products of the historical and cultural precipitation of different regions and different countries [3].

As a cultural form, clothing runs through the history of various periods in the East and the West. In the long process of human history, Chinese clothing and Western clothing have embarked on different development directions because of different aesthetic consciousnesses. However, in the long history of development, Eastern and Western clothing and clothing also have the convergence and integration of styles from time to time, and with the development of economic globalization, the trend of integration of Chinese and Western costume culture is also strengthening. While discussing the cultural differences between Chinese and Western costumes, we should also think about the importance of maintaining national characteristics under the impact of globalization. Therefore, it is of great significance to explore the differences between Chinese and Western costumes.

## 2. State of the Art

“Appearance” is an important part of nonverbal communication in intercultural communication [4]. People will consciously or unconsciously spread a lot of information to the outside world through clothing, makeup, ornaments, and other things, and from different costumes, it reflects the different aesthetics of China and the West, but because of the different aesthetics of China and the West, the difference in clothing is determined.

So what is the difference between Chinese and Western aesthetics? From the perspective of traditional Chinese aesthetics, Chinese emphasizes the beauty and elegance, and embodies the unique outlook on life and aesthetics of life settling down, returning to the heart, experiencing all things, connecting with heaven and earth, integrating self and all things as one, and obtaining the soul' Chinese suitability [5]. Therefore, in terms of clothing Chinese love, a low-key and elegant feature, outstanding but not ostentatious, gorgeous but not gorgeous [6]. And Westerners due to the characteristics of the living environment near the sea, love a kind of innovation and personality, they advocate freedom and dreams, so in the choice of clothing also reflects their exaggerated, distinctive characteristics, often in the mix-and-match, hip hop, rock and roll, and even a peculiar Gothic style appears, but the daily clothing fully reflects their debauchery, more emphasis on the comfortable, simple and decent characteristics of clothing [7]. In addition, China and the West also hold different views on “beauty”: many countries in the West generally do not deliberately comment on the natural appearance of others, even if they praise the natural beauty of others will make people very uncomfortable, but they tend to praise others' modified appearance, such as makeup, hairstyles, clothing, accessories, and so on [8]. This is because in the traditional Western aesthetic thought, artistic beauty and artificial beauty are regarded as higher realms than natural beauty, as Hegel clearly said in “Aesthetics”: “We can definitely say that artistic beauty is higher than natural beauty.” Because artistic beauty is produced and regenerated by the mind, the mind and its products are much higher than nature and its phenomena, and artistic beauty is much higher than natural beauty [9]. The Chinese is very different, Chinese generally believe that the natural beauty of “natural beauty” is more praiseworthy and flattering than the artificial beauty and decorative beauty after makeup, so when commenting on the appearance, Chinese like to evaluate a person's natural appearance, thinking that praising a person's natural beauty can make the other party happy and feel respected, so since ancient times, there is a kind of “clear water out of the hibiscus, natural to carve” saying. In addition, Chinese generally believe that plain face is more beautiful, is the beauty of “grass color remotely look close but nothing,” and the most advocated plain face clothing, and Westerners' preferences are very different [10].

### 2.1. The Characteristics of Traditional Chinese Costumes and Cultural Concepts

1. Be Good at Expressing the Subtlety of Form and Color
2. Hazy, hidden but not revealed, implied allegory, giving people an aesthetic feeling. This kind of subtlety is sometimes displayed through style, and sometimes it can also give people the beauty of overall harmony through modeling, layout, color, line, and other means.
3. Pay Attention to fine Artistic Techniques and Craft Expression
4. A large number of embroidery, streamers, patterns, and other decorative techniques are used to express rich imagination and achieve realism with romantic atmosphere.
5. Pay Attention to the Atmosphere Effect of Style and Stability
6. The overall coordination of clothing gives people a sense of order and harmony and beauty, serious and solemn, beautiful and elegant, can play a role in foiling, clothing culture and environment to match, more distinct atmosphere of the times.
7. Pay Attention to the Nationality of Clothing Culture
8. Costume culture is one of the important symbols of a nation's personality and national characteristics. As a folk phenomenon, clothing has a distinct national character. Long-term exchanges between different ethnic groups, Clothing cultures influence and infiltrate each other, and even intentionally borrow and imitate. But the Chinese nation has its own aesthetic tastes, ethics and cultural concepts, so it has its own dress code.

### 2.2. The Characteristics of the Cultural Concept of Western Clothing

1. Advocate human body beauty
2. From ancient Greek times to the present, Western art, including clothing, often regards the praise of praise and the display of the natural beauty of the human body as supreme models. As a result, clothing has become a “by-product” on Westerners: women show the beauty of their bodies by exposing or hanging silk, while men show the health and strength of their skin more nakedly.
3. Clothing is to attract the attention of the opposite sex to themselves Western clothing through the human body curves and some sensitive parts of the nudity treatment, to maximize the attractiveness of clothing, to give people an indescribable sense of beauty, in order to produce.
4. Psychological effects make people quickly enter the pure aesthetic realm.
5. Highlight personality
6. Westerners dress heavily on self-expression and the pursuit of individuality. Seeking a breakthrough in balance and one-sided excavation, self-design, self-expression, self-creation and unique; through dress, fully indicate the ideal realm of the self and various concepts, show self-worth, so as to mark the self.
7. Pursue sensory stimulation
8. Western clothing focuses on enabling the viewer to inspire sensuality and form unusual sensory stimuli. Through careful design, unique color combination and special line segmentation, the design master fully reflects the psychological and physiological characteristics of gender. So, in the West, sexy clothing is the main factor defining the success of its brand designers.

## 3. Methodology

### 3.1. Archaeological Connotations of Knowledge

Michel Foucault proposed this method of analysis in The Archaeology of Knowledge. Knowledge archaeology refers to excavating like archaeology, deeply studying things that are unfamiliar to our cognition, and reinterpreting the things that we think we know [11]. Knowledge archaeology is different from the historical research we usually use, it is actually to abandon our existing, known things, to redig and explore, in the existing knowledge space to find those hidden in the depths of time of historical clues, in simple terms, knowledge archaeology is a kind of knowledge reunderstanding, is to restore the original appearance of things on the basis of its examination, screening, identification, search for its roots, is to open up the “known” in-depth study as shown in Figure 1 [12].

### 3.2. The Main Manifestations of the Similarities and Differences between Chinese and Western Clothing

In China's 5,000-year history, there is a rich and long history and culture, and there are great differences between traditional Chinese culture and the fast culture spread in the West, of course, there are similarities between them. Studying, “archaeology” the history of the development of Chinese and Western clothing, and observing the Chinese and Western clothing we see now, we can find that there are many differences and similarities between them from the aspect of clothing design alone. The similarities and differences between Chinese and Western costumes are inseparable from Chinese and Western cultures, because the differences between Chinese and Western cultures make their forms of expression different, and because the commonalities between Chinese and Western cultures make them similar. Culture is not good or bad, and there is no high or low clothing as shown in Figure 2 [13].

### 3.3. Differences in Clothing Colors

Color plays an immeasurable role in the aesthetics of clothing; it is an indispensable part of clothing, but also an indispensable part of people's lives. Studies have shown that people's sensitivity to clothing color is greater than people's sensitivity to the shape of clothing, so color has a very important position in clothing. People's most primitive instinct is to decorate clothing with color, which also shows the importance of color in clothing for people. “The color of Chinese clothing is more ethical, requiring clothing to maintain social order; the color of Western clothing is more emotional, and attaches importance to the regulation of people's psychology by clothing [14].”

This is because Chinese value the whole, while Westerners care about the individual. Chinese focus on the whole and ethics, while the West cares more about what the individual wants as shown in Tables 1 and 2. Therefore, the difference in the choice of clothing color can reflect the difference between Chinese and Western cultures [15].

In China's thousands of years of history and culture, it can be found that the choice and love of the color of Chinese clothing is inseparable from China's long-standing traditional culture. The preference of a nation or a country for color actually reflects the intrinsic culture of this nation and country. In ancient China, the color status of traditional clothing was influenced by the five elements of yin and yang, which defined the five colors of blue, red, black, white, and yellow as the five colors corresponding to gold, wood, water, fire, and earth, respectively, and promoted them as positive colors Other colors other than these five colors are derogatorily referred to as interchromatic [16]. In the early days of ancient China, people believed that black was the color that dominated all things, and it was the symbolic color of the gods, and history recorded that black was precious during the Qin Shi Huang period, and the clothes worn by Qin Shi Huang were mainly black. Red is also loved by many people in China, Chinese believe that red represents auspiciousness and festivity, and the walls of the Forbidden City are mostly red. According to historical records, the Jin Dynasty implemented the Jinde system, with red as the most expensive, so the Emperor of the Jin Dynasty wore red robes as shown in Figures 3 and 4 [17].

Chinese part of the admiration for yellow comes from the worship and reverence for nature in the early days of ancient China, and it is recorded in the Zhou Yi that yellow is the color of the central soil in the Five Elements Science, so in that period yellow was called zhengse, the most important color. The Chinese nation originated from the Yellow River region, the yellow land is the original habitat in ancient times, because yellow is the color of the earth, so people have a sense of reverence for yellow, but also because of the worship of the earth, gradually produced the idea of yellow as the respect. The other part was inextricably linked to the royal nobility during the feudal period. During the Sui Dynasty in ancient China, emperors began to wear yellow robes, and Tang Gaozu stipulated that “hundreds of officials and people are not allowed to wear yellow clothes,” and yellow became the color used for the emperor, in addition to symbolizing that the Chinese dragon is also yellow. Chinese gave yellow a symbol of centralized power, and during the feudal imperial period, yellow was the color used by the royal court and was a representative of power. Because of this power effect, yellow has gradually become the most popular color of the Chinese nation [18].

The positive color was generally loved by the royal and high-ranking dignitaries, and slowly the positive color evolved into a symbol of power. It is not difficult to see that the choice of color in China's clothing has been influenced by China's traditional feudal etiquette culture, and positive color has gradually become the color that people love and pursue in color matching. China's feudal hierarchy was strict, the royal aristocracy was extremely high, and the imperial power was supreme. We can clearly find from the color of clothing: any color that is favored by the royal nobility is forbidden to be used by the people, and if it is violated, it will lead to the disaster of killing. Conversely, if a color is abandoned by the royal family, then the color will also be regarded as a despicable color by the common people. To sum up, in ancient China, the choice of clothing color came from the submission to the feudal etiquette system, and the common people had a reverential and yearning heart for the right color [19].

In the West, Westerners' choice of color comes from individual emotions. They believe that color is the embodiment of emotions, they tend to make choices according to their own specific characteristics, they pay more attention to the individual, and most of them are not bound and agreed by the ruler in the choice of color. Westerners believe that color also has feelings, is the carrier of their emotions, just like the mirror of their own heart. In Roman times, white and purple were loved by Westerners. They believe that white is a symbol of purity and beauty, which cannot be defiled and violated, which is one of the reasons why until now Westerners generally choose holy white as the main color of wedding dresses [20].

It should be noted that purple, due to the complexity of the production of purple dye, purple is very scarce, usually only appearing in the rulers of the country and the royal family. Similar to ancient China, purple was only used for national rulers, symbolizing noble emperors, which was also a manifestation of a high degree of centralization. But this is not evident in the West as in China. During the Renaissance, due to the emergence of humanistic ideas, people's choice of color became more and more bold, and the variety of choices was also increasing. For example, in France, people like to decorate clothes with white, lilac purple, rose powder, and sky blue; in Spain, people worship gray and rose red; in Britain, black is sought after by the British, black is mysterious and noble in the eyes of the British, and black is sometimes chosen for formal occasions such as funerals. Westerners choose the color of clothing mainly related to their own collocation, preferences, and their hearts, sometimes they will use warm red to express their inner pleasure at that time, sometimes they choose black to attend important occasions to show their attention to it. Westerners choose color from within themselves, and unlike China, they are most often unconstrained by other conditions.

### 3.4. Differences in the Appearance of Clothing

Traditional Chinese clothing is more about visually highlighting the longitudinal effect, and designers usually use sagging lines to show the overall slender feeling. In traditional clothing, the barrel-shaped robe skirt is combined with the long sleeves that can cover the hands, and the design of the shoulder design is relatively subtle, not exaggerated, and does not pay attention to emphasizing the shoulder line. Traditional Chinese clothing forms used to be open in the form of plackets and plackets, which were mainly two styles. Traditional Chinese clothing usually adopts the two basic forms of tops and bottoms and clothes, which intersect in China's thousands of years of history and culture, are compatible and inclusive, and cover a wide range. Traditional Chinese costumes are more subtle and restrained than Western costumes; in fact, these forms of expression are inseparable from traditional Chinese culture. Chinese dressed in clothing to pay attention to subtle beauty, relatively conservative, very restrained expression of personality. Traditional Chinese costumes attach the same importance to the expression of imagery and care about artistic conception as the famous Chinese landscape paintings, just like the poem “Thousands of calls begin to come out, like a pipa half covered,” traditional Chinese clothing pays attention to vague and subtle beauty. Although this kind of loose, unsuitable clothing cannot outline the human body lines and beautiful human contours, this kind of elegance that hides the curvy beauty of the human body is not a different kind of beauty.

Traditional Chinese clothing hides the human body and never exposes half of the skin. The clothing emphasizes loose, unsuitable, overlapping underwear outerwear, layer after layer like a lampshade covering the human body. Compared with Western clothing, traditional Chinese clothing is dull, bulky, and inconvenient. Westerners pay attention to human aesthetics, they dare to express themselves, dare to show their beauty, they are different and different, so Western clothing is more “bold and wild” compared with traditional Chinese clothing. Westerners attach importance to the curved beauty of the human body, so Western clothing is mostly to highlight the curves and human body lines. The evolution of Western clothing styles began with the wrapped style in ancient Greece and ended with the wrapped unformed clothes and the semimolded clothes in the front opening type in the Middle Ages. Unlike traditional Chinese clothing, traditional Western-style clothing attaches importance to the visual sense of transverse in appearance. Traditional Western-style clothing often uses a horizontally expanding shoulder contour to achieve a visual lateral impact. Western designers like to use hard collars, inflated, and exaggerated sleeves to achieve the effect of radiating outwards.

Compared with traditional Chinese clothing, Western traditional clothing design is more open, exaggerated, and has ups and downs. Of course, not all Western-style clothing advocates tightness and revealing, and some Western-style clothing also pays attention to cover—Western traditional clothing also has wrapped styles. This kind of clothing is three-dimensional cut, emphasizing a close fit with the human body, in order to achieve the effect of outlining the perfect curve of the human body and fully highlighting the body shape of the human body. The shape of Western-style clothing, whether exposed or wrapped, is for one purpose—to highlight the human body line, pay attention to, and advocate the beauty of the human body. From a structural point of view, whether it is a robe, a shirt, a shirt, a gown, or a gown, there is usually only a structural line connecting the seam of the sleeve and the side hem. Traditional Chinese clothing adopts the traditional Chinese flat straight line cutting method, without shoulders and armholes, flat on the ground as smooth as paper, emphasizing the loose and comfortable dressing experience. Western clothing mostly uses three-dimensional tailoring methods to achieve the effect of matching the three-dimensional human body; this three-dimensional cutting method treats the human body as a three-dimensional polyhedron, using pleats and provincial processing and other clothing processing means, carefully considering the convex and convex, and undulating relationship of the human body from top to bottom, from front to back, which is a more humane cutting method. Traditional Chinese costume culture pays more attention to the expression of imagery, using the cutting method of flat lines and curves to make the clothes comfortable and not completely fit the body. Traditional Chinese clothing is not nude, not ostentatious, does not highlight the lines, and implicitly shows the smooth and gentle, warm, and flowing curved beauty of the human body in the vagueness of the covering. The modeling consciousness of traditional Chinese clothing is rhythmic, and the human body exudes a high-level line beauty between loose and unclothed clothes and walking, which is a subtle and intriguing beauty, which is different from the direct expression of the West. China's traditional clothing space modeling is expressed through the rhythm of “virtual and real” and “light and dark.” Western clothing culture gradually sprouted the seed of spatial consciousness after the Middle Ages. This reflects the Westerners' search for space and their desire to occupy more space, so Westerners like to increase the volume of clothing, such as filling clothes with items, and so on. They use clothing as a tool to expand and take up more space.

This exaggerated clothing shape keeps a certain distance between people and nature, between individuals and people, and between individuals and the whole. From the western people's clothing space modeling, it reflects the western people's cosmology, and also reflects the opposition between man and nature, mind and environment, subjectivity and objectivity. Due to the different philosophical and aesthetic concepts of the East and the West, different shapes are reflected in the clothing, and they also reflect completely different spiritual charm and cultural connotations. In traditional Chinese social and family education, clothing codes of conduct are regarded as one of the important contents of self-cultivation, which has long affected the Chinese people's hobbies and lives. Chinese pay more attention to the content of morality and ethics in terms of dress, and use clothing to cover up human beauty and not expose, so as to meet the moral requirements of Confucianism.

Traditional Chinese clothing pays attention to the beauty of people's spirit, temperament and charm, and does not emphasize highlighting the body but cares about the inside. Western clothing culture is diverse; it is all-encompassing, accepting all personalities. In summary, it is not difficult to see that under the influence of different cultures, the expression of clothing is different. The differences in style and appearance between Western and Oriental clothing are also closely related to the cultural background. Traditional Chinese feudalism, especially in women's clothing, is particularly evident. Western ideas are open, personality differences are prominent, and Westerners are innovative in the way they wear clothing and pursue individuality. Western culture is open and all-encompassing, and all “strange” things in the West are acceptable and accommodated, which is greatly reflected in the various costumes of the West. Western costumes take a variety of forms and are dazzling, such as the aristocratic Gothic style, the gorgeous Rococo style, the richly varied Romantic style, the gorgeous and subtle Victorian style, and so on. These exquisite and individualized Western costumes reflect the Pursuit of Individuality by Westerners.

### 3.5. Differences in Clothing Patterns

In the choice of patterns, Chinese and Western clothing also shows completely different and distinctive choices. In China, whether it is ancient or modern, whether it is aya silk or burlap, we can see patterns that symbolize auspiciousness. Chinese like to express their worship and admiration for totems by choosing patterns on the decoration. In China, patterns such as dragon and phoenix chengxiang, nine dragon play beads, and magpie dengmei are usually chosen to express the hope of a happy life. In China, we often use the pattern symbolizing good wishes on clothing, which is our good wish and a kind of expectation and desire for auspiciousness. The hierarchical identity of the decorative patterns of Ming Dynasty clothing reflects the “Taoist” spirit of Chinese's pursuit of a high degree of unity of form and content in the aesthetics of decorative design. The evolution of patterns on Western clothing is also constantly changing. During the Italian Renaissance, people liked to use floral patterns on clothing; during the Louis XV period, due to the influence of the Rococo style, Westerners liked to use S-shaped or curved vine patterns; while modern Westerners popularly chose Fauvist patterns.

### 3.6. Differences in the Performance of the East and the West in the Shape Structure

The aesthetic concept of Chinese clothing is expressed in the shape of the structure of the image, this kind of flat straight line and curve cutting method makes the clothes fit and not completely fit, not nude and publicity, not to try to bind, in the shape does not show the three-dimensional relationship with the human body. With this kind of flat cutting method without clear convexity, a white texture and harmonious and unified space shape were obtained. This kind of flat cut clothing style tends to be more holistic, and the Chinese-style wide clothes are as flat as the scrolls and fabrics when placed or hung, and their generosity and openness when dressed are clear at a glance (see Figure 5). The aesthetic characteristics of Chinese-style clothing reflect the aesthetic aspirations and cultural characteristics of the Chinese nation.

Chinese influenced by the complementary aesthetic ideas of Confucianism and Taoism attaches importance to the combination of reason and reason, pursues leisure, blandness, moderation, and pursues spiritual meaning beyond the body. The shape of traditional Chinese clothing emphasizes the longitudinal feeling, often sagging lines, long sleeves over the hand, barrel-shaped robe skirts, and vertical decorative techniques, making the human body appear slender. The costume is relatively fat, and the cuffs and hems have a wide sagging tendency. The slenderness of the shape of the costume compensates for the relatively short figure of the Orientals, produces optical illusions in the senses, and achieves perfection and harmony in proportion. The smooth shape of the garment matches the softer contour lines of Chinese's face as shown in Figure 5.

Due to the continuation of ancient Greek and Roman cultures and the intersection and fusion of classical, Christian and Germanic cultures over the centuries, clothing has moved from a loose style to a composite style. That is, the clothing structure has undergone a process from simple to complex, from flat to three-dimensional. This three-dimensional form has been maintained and continued for thousands of years in the history of Western clothing, so that the Western clothing form has become a shape based on plastic, and strives to express the three-dimensional cutting method of the human body, whether it is hung in the closet or worn on the body, or walked up, always maintaining a relatively static three-dimensional geometric space effect. This reflects the Westerners' exploration of space, with an obvious psychological motivation of “self-expansion,” increasing the volume of clothing shapes, eager to occupy more space, and regarding clothing as a tool to expand their own body shape. This exaggerated costume shape maintains a certain distance between people and the whole of nature, and between individuals and people, reflecting the cosmology of Westerners, but also reflecting the opposition between man and nature, mind and environment, subjectivity and objectivity. Especially after the Renaissance, clothing has been developed in a tortuous way again and again in the transition from natural shape to peak decoration and exaggerated shape. The different cultural backgrounds and aesthetic concepts of the East and the West have formed different ways of modeling in the clothing, reflecting different spiritual charms. With the development of today's economic globalization, the trend of integration of Chinese and Western costumes and cultures has also been strengthened as never before. Chinese clothing is also constantly in line with the world, traditional clothing design is gradually integrated into the Western fashion elements, while Chinese elements are also affecting the development of the international fashion industry. Although the Eastern and Western people have different shapes and concepts, it is the same desire to pursue the artistic conception of truth, goodness, and beauty in clothing. Today's clothing design to express the spirit of the times is to let the national spirit integrate into the world spirit, let the ancient spirit integrate into the future spirit, so that the different spirits and charms expressed in the background of different philosophies and aesthetic concepts in the East and the West complement and strengthen, so as to achieve the commonality of the mind and thought, so as to overflow with new spirits and concepts, and convey the inner charm of the atmosphere of the times.

### 3.7. Differences in Dress Styles in Chinese and Western Costume Cultures

Whether it is Ancient Chinese clothing or modern clothing, they are mainly under the upper and lower clothes, and they all follow the design style of opening and closing. In ancient times, clothes were mainly fixed by ropes and straps, and consisted of many robes. In the process of wearing, first wear a top, then a bottom, first a shirt, and then a layer of outerwear. Since modern times, China's clothing has become more and more frequent and simple, although it has also been impacted by foreign clothing culture, resulting in different closure designs such as dresses and sweatshirts, but in general, most of them still follow the style of opening and closing before and after, tops and pants.

Western clothing is divided and composed of multiple parts, so it is necessary to wear a underwear with a fixed effect first, and then wear various parts of the clothing according to the curve of your body. From the perspective of closure, Western clothes are mostly front closed and back open, and the elasticity of clothes is adjusted through the back rope. This closure has also continued into modern Western clothing design, such as cross-head dresses and sweaters.

The implicit and freehand nature of Chinese clothing and the directness and realism of Western clothing show two completely different philosophical views and values, which also forms a completely different aesthetic, which is manifested in the tailoring of clothing, and forms two distinct systems, namely the Chinese clothing culture system centered on straight line cutting and the Western clothing culture system centered on curve cutting. The former has created a “natural” and “flat” clothing form; the latter has created a “human,” “three-dimensional” clothing form. The former is “made in one go,” fully maintaining the original appearance of the cloth, the structure is very concise, is “nonconstructive”; the latter is based on the shape of the person to “disintegrate” the clothes, divided into several independent parts, respectively, after completing the shape of these parts and then assembled, the structure is complex, is “constructed.” The former fully respects the existence of people, clothing modeling depends on the human body to complete its final shape, the degree of molding is low, mostly belong to the “semi-formed class”; while the latter often ignores the existence of people, the clothes themselves are a kind of “humanoid” “shell,” many times it is forced to adapt to this artificial “shell,” its degree of molding is higher, mostly belong to the “molding class.”

## 4. Result Analysis and Discussion

### 4.1. Analysis of Characteristic Factors of Contemporary Chinese-Style Clothing

#### 4.1.1. Questionnaire Design

In view of the recognition of Chinese and Western Chinese-style clothing, this study conducted a special survey, of which the questionnaire contains two main parts, first, mainly to learn the basic situation of the respondents and the basic understanding of Chinese-style clothing, such as gender, age, occupation, education level, personal monthly income, and whether the respondent has seen Chinese-style clothing, what Chinese-style clothing has been contacted; second, first, through the collation and summary of a large number of Chinese-style clothing design literature, and then by expert argumentation. Finally, through the identification of Chinese-style clothing elements in the 100 cases of pictures, and the analysis of the main constituent factors in the process of realizing the design of Chinese-style clothing, the materialization factors and social factors affecting Chinese-style clothing were extracted, of which 26 materialization factors were extracted, including embroidery, hand printing and dyeing, paper cutting, hand-painted ink, belly pocket, standing collar, placket, shoulder seam, slit, disc buckle, brocade, cyan, red, yellow, white, black, green, purple, and planting object patterns, animal patterns, character patterns, Chinese character patterns, geometric patterns, blue and white porcelain patterns, tassels, and Chinese knots; four social factors: practical value, aesthetic value, humanistic value, and social value. Then, the “Five Point Scale” of Li Kete was applied to the above 26 materialization factors and 4 social factors to develop a questionnaire, and the participants evaluated the importance of each index according to their cognition of Chinese-style clothing, thereby determining the recognition of each element in the characteristics of Chinese-style clothing factors.

The respondents' basic situation table reflects that the randomness of sample collection is relatively ideal. The Chinese and Western respondents basically included people of different genders, different ages, different occupations, different academic qualifications, and different monthly incomes.

Among them, as shown in Figure 6 the proportion of men and women in China is basically the same, with men accounting for 45%; from the perspective of age structure, it is mainly under 25 years old, accounting for 76%; from the perspective of occupational composition, students account for the largest proportion, 74%; from the perspective of academic structure, bachelor's degree and above account for the largest proportion, a total of 86%. “Among them, undergraduates accounted for 72%; from the perspective of monthly income structure, it was mainly below 2,000 yuan, accounting for 59%, which was mainly related to the respondents as students. The proportion of men and women in foreign respondents is basically the same, and there are slightly more women, accounting for 64%; from the perspective of age structure, it is basically distributed between 25 years old and 26–30 years old, accounting for 43%, respectively. With 31%; from the perspective of career level, the proportion of students is the largest, 64%; from the perspective of academic distribution, bachelor's degree and above account for the largest proportion, of which undergraduate is 50% and master's degree and above is 29%.” From the monthly income structure, the ratio of each level tends to be balanced, of which 23% is less than 2000 yuan, and 17% is 17% of 2001–5000 yuan. 5001–10000 yuan accounted for 36%. About 10001–50000 accounted for 20%, more than 50,000 yuan accounted for 4%. Since the attention to clothing is concentrated in women, young and middle aged, highly educated, and middle class, therefore, the selection of domestic and foreign samples has a certain rationality.

#### 4.1.2. Questionnaire Recycling Analysis

In order to obtain the basic understanding of Chinese and Western style clothing, the questionnaire identified the question “Do you think there is a Chinese-style costume in contemporary times?” “9% and 17% of people outside China and the West believe that there is no Chinese-style clothing, so the subsequent analysis cannot be included in the statistics, so the real effective questionnaire is 197 in China and 58 in the West.”

It can be seen that 6% of people in China believe that they have no understanding of Chinese-style clothing, 69% of people think that they do not know much about Chinese-style clothing, and 24% think that they know only 1% about Chinese-style clothing.. It can be seen that most people in China think that they do not know much about Chinese-style clothing; 14% of people in foreign countries (in the West) think that they have no understanding of Chinese-style clothing, 52% think they do not know much about Chinese-style clothing, and 27% think that they know little about Chinese-style clothing, and 7% of people think they know all about Chinese-style clothing. About 75% are completely unknown and poorly understood at home, 67% are foreign, 25% are understood and fully understood domestically, and 1% are foreign. It can be seen that the degree of understanding of Chinese-style clothing is similar in China and in the West.

It can be seen that the degree of recognition of Chinese-style clothing in China is higher than that of Western countries, of which 91% of people in China believe that there is a Chinese-style clothing, and only 83% of people in the West think that there is a Chinese-style clothing; 90% of people in China think they have seen Chinese-style clothing, and only 76% of people in the West think they have seen Chinese-style clothing; 81% of people in China like Chinese-style clothing, and 79% of people in the West like Chinese-style clothing, which is the same as in China; for whether Chinese-style clothing is needed, The difference between home and abroad is relatively large, 93% of people in China think that they need Chinese-style clothing, while only 60% of people in the West need Chinese-style clothing; but the proportion of Chinese-style clothing in the West is 36%, while the proportion of domestic purchases of Chinese style clothing is 30%, lower than abroad.

Through the questionnaire setting, the identification of Chinese and Western social general groups in Chinese and Western society whether Chinese-style clothing is suitable for the popularity of contemporary clothing, and whether Chinese-style clothing needs to be improved and progressed, so as to provide reference for Chinese-style clothing to better adapt to Chinese and Western clothing fashion.

## 5. Analysis of the Reasons for the Difference between Chinese and Western Clothing

The Chinese nation's thousands of years of history and culture contain a profound costume culture, under the accumulation of these historical and cultural precipitations, China's unique aesthetics and clothing forms have been formed, and Chinese clothing emphasizes more on “the unity of things and me,” which is contrary to the West. Western clothing culture emphasizes the separation of subjectivity and objectivity, believing that “things” and “I” are opposites. Therefore, traditional Chinese clothing is mainly based on wide clothes, while the West is mainly based on clothes that outline the beauty of human lines. The difference between Chinese and Western clothing isactually the difference in moral concepts between Chinese and Western cultures. In essence, the cultural differences between China and the West are essential. The Chinese culture is the overall culture, while the West is the individual culture. In terms of thinking, the Way of Thinking of Westerners is partial and polarized. And Chinese way of thinking is holistic and impartial. In terms of personal values, Westerners focus on the self, they are the center of everything, and everything revolves around themselves.

Westerners believe that there is an individual who has a society, that he himself is the foundation of the whole society, and that the individual is higher than the whole. Chinese values emphasize the whole, and personal interests are subordinated to the interests of the whole, with the whole as the core. Because of different cultural and historical environments, the moral concepts of Westerners in culture are in stark contrast to the moral concepts of our Chinese culture.

The moral concept of Chinese is based on the composite social ethics and moral code of conduct established by Confucian and Taoist culture, including the moral thought of Taoism, the promotion and restraint of Confucian moral principles such as benevolence, righteousness, wisdom, loyalty, and benevolence. These are moral concepts unique to Chinese. These moral concepts and norms have effectively maintained the stability of the social system and society. The Western moral concept is based on ancient Greek philosophy and Christianity, and the establishment of its moral concept from the aspects of cultural traditions, economic structure, political system, and interpersonal relations makes the modern Western ethical and moral system manifest as an ethical system of active external seeking. Western morality is mainly manifested in: the pursuit of individualism, advocating freedom, daring to take risks, honesty and extroversion, frankness, and straightforwardness. Therefore, the differences between Chinese and Western clothing are inseparable from their culture.

## 6. The Fusion of Eastern and Western Costume Cultures

As a cultural form, clothing runs through the history of various periods in the East and the West. In the long process of human development, Chinese clothing and Western clothing have embarked on different development directions because of different aesthetic consciousness. Chinese clothing culture pays attention to the pursuit of the spiritual level, and the clothing style is relatively conservative, showing a dignified, elegant and subtle oriental atmosphere. Western clothing culture pays attention to the pursuit of scientific level, and the pursuit of clothing styles is attached to the wearing of human forms, so the curve of clothing is obvious, showing the beauty, boldness, and elegance from practicality. However, in the long history of development, Eastern and Western clothing has also had a convergence of styles, especially since the successive changes in Eastern and Western clothing in the early 20th century, this integration has affected the development of the entire social clothing style: Oriental clothing has absorbed the three-dimensional cutting method of the West, making the clothing close and lightweight; the West has abandoned the distorted human beauty and liberated women from the corset that damages health. Moreover, in order to adapt to life, both the East and the West have changed the tedious decoration and clothing structure. With the development of today's economic globalization, the trend of integration of Chinese and Western costume culture has also been unprecedentedly strengthened. The Chinese garment industry is striving to integrate with the world, take a fashion plus national characteristics road, and integrate Western fashion elements into traditional clothing design, while Chinese elements are influencing the development of the international fashion industry. In the 20th century, when the French costume designer Yves Saint Laurent held a retrospective exhibition of his works at the National Art Museum of China, he said in the preface: “We Westerners have received a lot from China!” And modern Western designers are increasingly borrowing and applying Eastern and ethnic elements in their designs. China is an ancient country with a history of 5,000 years of civilization, as a garment worker should “use foreign for Chinese use,” learn from the Western costume culture, so as to develop its own national costumes. While discussing the cultural differences between Chinese and Western costumes, we should also think about the importance of maintaining national characteristics under the impact of globalization. Therefore, it is of great significance to explore the differences between Chinese and Western costumes.

## 7. Conclusion

In ancient China, clothing was often seen as a manifestation of power and status. As a country of etiquette, China attaches great importance to etiquette and system, and the clothing of Chinese is the external expression of etiquette culture. Traditional Chinese clothing pays attention to the “unity of heaven and man” in design, emphasizing the inner pursuit. Traditional Chinese clothing follows a law and a norm, which is a “Taoist” aesthetic. The clothing culture of Westerners is very different from that of China, and the West advocates human beauty and requires clothing to better outline the beauty of the wearer's body and lines. In the eyes of Westerners, the human body line is beautiful. Therefore, the aesthetic design of clothing requires that the shape of clothing and the wearing of clothing can fully and perfectly reflect the beautiful posture of the human body, which can be said to be a “humanized” aesthetic concept. The difference between the aesthetic concepts of “Taoization” and “Humanization” in Chinese and Western clothing design has been reflected to varying degrees in the clothing design of various dynasties in China and the West for thousands of years. This study compares the aesthetic concepts of Chinese Design in the Ming Dynasty and the Western Renaissance in the same period from the three aspects of clothing, color, and decoration, and the difference between this kind of “Taoization” and “Humanization” can be seen slightly.

From the perspective of intellectual archaeology, why should we study the cultural differences between China and the West? Because the differences in Chinese and Western clothing are influenced by culture. In the past, when we discussed clothing, we chose to do a specific content description, using the same or different statements to summarize and express, but we may ignore the exploration of the essence of culture. Because the reason for understanding the differences between Chinese and Western clothing is to explore the cultural differences between China and the West, not only those specific meanings that seem to have been summarized by predecessors, but also a lot of deeper logic, meaning, and discourse expression behind them, which need to be further explored.

With the development of economic globalization, the trend of combining Chinese and Western costume culture will gradually strengthen, before we learn from the Western costume culture, the first thing to do is to continue to add the inheritance of China's traditional costume culture, take its essence, remove its dross, innovate, and innovate, so that the excellent traditional Chinese culture can be continuously circulated. Combine it with modern design concepts, learn the humanistic concept of Western clothing, and combine the two to make our Chinese clothing culture develop better.

## Figures and Tables

**Figure 1:** The representative of oriental clothing—cheongsam.

**Figure 2:** Clothing styles in the middle ages in Europe.

**Figure 3:** The subtlety of shape and color.

**Figure 4:** The unique artistic features of the east.

**Figure 5:** Costume modeling under the background of Chinese culture and western culture.

**Figure 6:** Analysis of different components at home and abroad to compare the situation of different respondents.

**Table 1:** Chinese clothing decoration overview.

Types	Jacket	Shirt	Coat	Robe	Vest
Quantity/piece	51	53	12	12	14

Form	Narrow long sleeves, long to abdomen; wide long sleeves or seven sleeves longer than buttocks	Narrow long sleeves, wide seven sleeves or long sleeves, as long as the abdomen or buttocks	Narrow long sleeves, short clothes, often only to the abdomen	9 men's robes, 3 cheongsam, narrow long sleeves	10 adult waistcoats and 4 children's waistcoats, 2 of which are draped

Collar type	No collar 2 pieces, vertical collar 49 pieces, collar height 3–8.5 cm	No collar 2 pieces, vertical collar 51 pieces collar height 3.5–7 cm	Stand collar, collar high 3.5–6. 5 cm	Vertical collar collar high: 4.5–6.5 cm	No collar 5 pieces, vertical collar, collar height: 3.5–7.5 cm

Door lapel form	32 right lapel, 18 left lapel, 1 right lapel	33 right lapels, 20 left lapels.	Opposite lapel	Right lapel	Right lapel 8 left lapel 1 opposite lapel 5

Sleeve type	Wide cuff width: 29–46 cm narrow cuff width: 14–18 cm	Wide cuff width 23–44 cm width of narrow sleeve: 12–18 cm	Cuff width: 15–25 cm	Cuff width 1 6–18 cm	Nothing

Decorative part	Lead edge, flap edge, sleeve edge, bottom pendulum, slit edge on both sides, edge insert, roll edge	Collar edge, flap edge, sleeve edge, bottom pendulum edge, roll edge decoration	Nothing	Women's cheongsam flap, collar edge, edge, men's robe undecorated	Flap, collar, edge, edge

Binding mode	A word buckle, disc buckle, hollowed out copper button	One word buckle, copper button, plastic button	One word buckle	One word buckle, gilded copper button	Disc buckle, one word buckle

**Table 2:** Western clothing decoration overview.

Species	Name	Quantity (piece)	Shape structure	Length (cm)	Waistline (cm)	Waist (cm)
Skirt	Horse skirt	47	On the basis of the traditional “apron” shape, with skirt door, pleated, beautiful dry, and so on, decoration, the skirt body is pleated on both sides, the middle part is the glossy surface, commonly known as the “horse face,” often decorated with embroidery or inlay, roll, collage lace.	88–96	43–68	11–16
	Phoenix tail skirt	27	Because the shape and phoenix tail is similar to the name, into a strip narrow type, the lower end decorated with moire, such as Italy grain and other auspicious patterns, some tail decorated with tassel, bell and so on, seen in etiquette and marriage occasions to wear.	82–92	43–51	10–17
	Pleated skirt	11	The pleated skirt or ichthyosis skirt retains the basic shape of the horse skirt and is embellished on both sides of the “horse face” with rich, fine, and neat pleats.	90–95	56–64	12–15

Pant	Crotch pants	18	Wide crotch, set waist, waist fat, wear the extra part of the waist to the middle fold, with a cloth belt to hold tight, foot edge decoration.	92–113	47.5–60	18–20

## Data Availability

The labeled data set used to support the findings of this study is available from the corresponding author upon request.
